# Sternal Metastasis of Lung Cancer: A Case Report and a Review of the Literature

**DOI:** 10.7759/cureus.51808

**Published:** 2024-01-07

**Authors:** Imane Legssyer, Oumayma Haloui, Siham Bouali, Afaf Thouil, Hatim Kouismi

**Affiliations:** 1 Department of Respiratory Diseases, Mohammed VI University Hospital, Mohammed First University, Oujda, MAR; 2 Department of Pulmonology, University Hospital Mohammed Vl, Oujda, MAR; 3 Department of Respiratory Diseases, Research, and Medical Sciences Laboratory, Mohammed Vl University Hospital, Oujda, MAR; 4 Department of Respiratory Diseases, Research, and Medical Sciences Laboratory, Mohammed VI University Hospital, Mohammed First University, Oujda, MAR

**Keywords:** sternal mass, squamous cell carcinoma, sternal biopsy, sternum metastasis, lung cancer

## Abstract

Primary sternal cancer is exceptionally rare. Secondary sternal cancer typically arises when cancer spreads either through the bloodstream from other sites or directly from neighboring lung or breast cancers.

Pain is the primary symptom, but these metastases can lead to skeletal-related events such as pathological fractures, hypercalcemia, and spinal cord or nerve compression, necessitating surgical or radiotherapy interventions. These events contribute to increased morbidity and costs for both patients and the healthcare system.

We report the case of a 63-year-old female patient who presented with a sternal mass and whose further investigations revealed metastatic lung cancer in the sternum.

## Introduction

Lung cancer is the second most common cancer, taking approximately 130,000 people's lives each year. One of lung cancer's challenges is that symptoms might be minor or nonexistent, resulting in many cases being discovered at an advanced stage of the disease. Metastasis in the chest bones may occur through two basic routes: hematogenous or lymphogenous [1].

Primary sternal tumors are uncommon, accounting for only 0.6% to 1% of all tumors. Furthermore, the vast majority of these sternal tumors are malignant [2].

Breast, lung, kidney, and thyroid cancers are common causes of sternal metastasis. Lymphoma, bronchogenic carcinoma, breast cancer, and pleural or mediastinal malignancies are all known to cause direct sternal invasion [3].

We present a case of sternal metastasis in lung cancer and a review of the literature.

## Case presentation

A 63-year-old man who had been a habitual smoker for six months arrived with many symptoms. A chronic dry cough, chest discomfort, dyspnea, and the presence of a tiny lump on the sternum were among the symptoms. These symptoms developed in the context of anorexia and weight loss.

A thoracic computed tomography (computed tomography) scan revealed an excavated lung mass in the right lingular region alongside an osteolytic lesion on the sternal manubrium. A fibroaspiration was performed to look for acid-alcohol-resistant bacillus [PRP1] [H2], and the results came back positive. Consequently, the patient was prescribed antituberculosis treatment.

The patient was referred to our department for further management due to the patient's deteriorating health and a noticeable increase in the sternal mass size.

During the general examination, the patient had pallor and asthenia; the vital signs recorded were as follows: a temperature of 37.8 °C, breathing rate of 20 cycles per minute, pulse rate of 100 beats per minute, and blood pressure of 100/70 mmHg.

During the inspection of the respiratory system, the chest was substantially enlarged in the sternal region. Palpation confirmed the existence of a 15-centimeter-long, hard, and heated mass. Inflammatory indications were present in the surrounding area, as well as two leaking ulcers (Figure 1).

**Figure 1:** Sternal mass measuring 15cm in diameter with inflammatory signs in the surrounding area, as well as the presence of two oozing ulcers (black arrows)

The thorax CT scan revealed that the appearance of the right lingular excavated lung mass remained constant. However, the size of the subsequent sternal osteolytic lesion increased. The lesion was now 6-9 cm long and had spread into the neighboring soft tissues (Figures 2-3).

**Figure 2:** Chest CT scan showing a sternal osteolytic lesion with a significant extension to the adjacent soft tissues (6x9 cm; white arrow)

**Figure 3:** Chest CT scan showing an excavated lingular lung mass (white arrow)

A second bronchoscopic examination was performed on the patient. During the inspection, a highly vascularized tumor mass was discovered obstructing the culmen of the left bronchial tree.

The immunohistopathological [PRP3] [H4] investigation of the bronchial biopsy re vealed a poorly differentiated squamous cell carcinoma in the bronchus (Figure 4).

**Figure 4:** Bronchoscopic image revealing a highly vascular bulge obstructing the culmen, which remains unremovable (white arrow)

Following the previous findings, an ultrasound-guided sternal biopsy was performed. According to the immunohistochemistry analysis, the biopsy results revealed a well-differentiated keratinizing and infiltrating squamous cell carcinoma.

The patient's final diagnosis was confirmed as squamous cell carcinoma in the right lung with metastatic tumors to the sternum.

The multidisciplinary team decided not to proceed with the resection. Instead, palliative chemotherapy was recommended as a treatment option. Unfortunately, the patient passed away before completing the first cycle of chemotherapy.

## Discussion

Although bones are a common site for lung cancer metastases, the sternum is rarely implicated, and only a few cases have been reported in the literature [4].

The pathophysiology of lung cancer bone metastasis can be divided into three stages: tumor invasion, tumor cell migration, and bone invasion. Genetic aspects, the microenvironment, and other adhesion-related factors may all affect it [5].

Clinically, sternal metastases are often asymptomatic; however, they may be revealed by pain or a bleedable sternal mass. Our patient had a sternal tumor that progressively increased in size [6].

The preferred imaging approach for assessing sternal lesions is a CT scan. It has advantages over radiography, particularly for identifying intrathoracic extent and mediastinal invasion. Furthermore, CT may help guide needle biopsy procedures. However, when it comes to determining mediastinal invasion, magnetic resonance imaging is considered to be superior to CT. Sternal metastases can take the form of lytic or sclerotic lesions. In this case, the lesion was osteolytic, extending substantially into the surrounding soft tissues [7].

Image-guided sternal biopsy has proven to be a reliable and safe approach to obtaining a conclusive histological diagnosis, regardless of the legion's specific characteristics or location. Our patient's diagnostic confirmation was obtained through an immunohistochemical study performed on an echo-guided sternal biopsy [8].

Metastases in the sternum are frequently treated with a combination of radiation, chemotherapy, and surgery. External radiation relieves bone pain, and sternal excision and reconstruction surgical procedures can treat primary sternal cancers and breast metastases. However, treatments for sternal metastases from lung cancer are limited, necessitating an individual approach. Palliative chemotherapy was chosen in this case because of the patient's deteriorating health [9-10].

## Conclusions

It is unusual for lung cancer to develop as a mass in the sternum, but medical practitioners must keep this possibility in mind when encountering a chest tumor, especially in patients who have a higher risk of lung cancer. This awareness is critical because early identification improves the prognosis and outcome for people diagnosed with lung cancer. By detecting the cancer early, healthcare practitioners can start immediate intervention and therapy, thereby increasing favorable outcomes and improving patients’ quality of life.
